# Titanium and titanium alloys in dentistry: current trends, recent developments, and future prospects

**DOI:** 10.1016/j.heliyon.2022.e11300

**Published:** 2022-10-28

**Authors:** Md Enamul Hoque, Nazmir-Nur Showva, Mansura Ahmed, Adib Bin Rashid, Sarder Elius Sadique, Tarek El-Bialy, Huaizhong Xu

**Affiliations:** a Department of Biomedical Engineering, Military Institute of Science and Technology, Dhaka, Bangladesh; b Department of Industrial and Production Engineering, Military Institute of Science and Technology, Dhaka, Bangladesh; c College of Information Technology and Engineering, Marshall University, West Virginia, USA; d Department of Dentistry & Dental Hygiene, University of Alberta, Alberta, Canada; e Department of Biobased Materials Science, Kyoto Institute of Technology (KIT), Sakyoku, Kyoto City, Japan

**Keywords:** Dental implant, Titanium alloy, Surface modification, Corrosion resistance, Osseointegration, Biocompatibility, Antibacterial activity

## Abstract

Many implant materials have been used in various dental applications depending on their efficacy and availability. A dental implant must possess the required characteristics, such as biocompatibility, corrosion & wear resistance, adequate mechanical properties, osseointegration, etc., to ensure its safe and optimum use. This review analyzes various aspects of titanium (Ti) and Ti alloys, including properties, manufacturing processes, surface modifications, applications as dental implants, and limitations. In addition, it also presents a perception of recent advances in Ti-based implant materials and the futuristic development of innovative dental implants.

## 1 Introduction

Titanium (Ti) and Ti alloys have increased extensively since the early 1980s. It has become the most accepted metallic biomaterial for its distinct properties and numerous biomedical uses (Özcan et al., 2012; Vizureanu et al., 2020; Takeuchi et al., 2020). Most of the time, metallic biomaterials are utilized for their high load-bearing capacity and fatigue strength to sustain the regular movements’ loads applied to them (Gegner et al., 2014). Titanium has been presented as one of the most encouraging designing biomaterials for its low modulus of elasticity, low specific weight, extraordinary resistance to corrosion, outstanding strength-to-weight ratio, good tribological properties, and exceptional biocompatibility (Hatamleh et al., 2018; Mutombo, 2018). Titanium alloys have the highest biocompatibility for biomedical applications than any metallic contents. However, because of the trend of osteogenesis, they are graded as bioinert materials compared to bioceramics like zirconia, alumina, hydroxyapatite, and combinations (Niinomi et al., 2008; Hoque et al., 2013, 2014; Ragurajan et al., 2018; Golieskardi et al., 2019). Current dentistry aims to reinstate the patient to usual purpose, health, aesthetics, and speech irrespective of the stomatognathic system's injury, atrophy, or disease. As a result, prosthetics in dentistry are one of the most excellent options for persons who usually are in appropriate oral health but have lost their teeth because of periodontal illness, an injury, or some other reasons (Oshida et al., 2010; Golieskardi et al., 2020). Many implants of many designs are now made from pure titanium and its alloys.

Until now, most metallic implants have been manufactured using traditional methods like hot rolling, investment casting, forging, and machining. However, numerous advanced manufacturing approaches are also utilized as all the implant alloys cannot be efficiently handled into the ultimate form in a similar method (Trevisan et al., 2017). Compared to traditional dental casting, titanium prostheses can be better made-up utilizing CAD/CAM (computer-aided design and computer-aided manufacturing) (Ohkubo et al., 2008). Nowadays, an innovative technique, 3D printing/Additive Manufacturing (AM), is customized to manufacture dental implants rapidly utilizing computer-aided design (Mohd and Abid, 2019). 3D printing/AM has demonstrated microscale resolution for the fabrication of implants through unclear efficiency of this process, but a potential approach for manufacturing dental implants (Thaisa and Andréa, 2019).

The metal ion release causes corrosion-related biological problems, such as toxicity, carcinogenicity, and hypersensitivity. The discharge of metal elements from the implant material to different body organs and peri-implant tissues was caused by biocorrosion, tribocorrosion, and their combination, which is a natural occurrence in the oral setting (Barão et al., 2021). While biofilms or high fluoride concentrations are existent, this effect is amplified. The presence of metallic particles activates T-lymphocytes, neutrophils, and macrophages, increasing the production of cytokines and metallic proteases. Furthermore, vanadium, aluminum, and Ti–6Al–4V particles are toxic and mutagenic, causing Alzheimer's disease, osteomalacia, and neurological issues (Kirmanidou et al., 2016). Ti and Ti alloys have noteworthy applications in orthopedics and dentistry. Hence, many implants are being introduced into the market daily. This review aims to determine why and how this material has progressed significantly, especially CAD/CAM. It is essential to study the interaction of Ti with the biological environment to decide what characteristics make this material and its alloys attractive as an orthodontic treatment material.

3D printing (3DP) is an emerging technology for dental implants, overcoming numerous dental difficulties, including diastema, crown damage, and tooth loss, because it plays a vital role in preventive/restorative dentistry. 3DP can attain close control of (i) multiple compositions, (ii) microstructure, (iii) mechanical attributes, and (iv) biological methods of attached tissues and organs with the implants. Indeed, it focuses on an exceptional attribution in dentistry for implant and restoration applications because of the significance of 3DP via CAD/CAM for manufacturing and implantation. It is plausible that Ti material with desired features for curing dental distortions increases the speed with lesser effort (Gagg et al., 2013; Unnikrushnan et al., 2021).

This study aims to describe the different uses of titanium and its alloys in Dentistry, along with its historical development, manufacturing procedures, and surface modification techniques. Various mechanical and physiological properties of Ti alloys are abridged in this review**.** It also discusses state-of-the-art and future perspectives about its utilization which will provide an overview for future manufacturers, researchers, and academicians.

## 2 Overview of commercially pure titanium (CP–Ti)

In 1791, Williams Gregor, a British mineralogist, discovered Titanium in Black Magnetic Sand' in Cornwall and termed it 'Menachite.' In 1795 it was rediscovered by a German mineralogist and scientific expert, Martin H. Klaproth, who named it Titanium. He deduced from the metal's properties that it was similar to the metal discovered by Gregor. An evacuee from Luxembourg, Dr. Wilhelm Kroll, is known as "The Father of the Titanium Industry." He introduced the Kroll, a useful Titanium production process. The US Bureau of Mines used the Kroll procedure to yield Titanium (Gosavi et al., 2013). The mechanical characteristics of CP-Ti (commercially pure titanium) are enumerated in Table 1 (Masa and Braunitzer, 2017).

**Table 1:** Mechanical properties of CP-Ti (Masa and Braunitzer, 2017).

Properties	Tensile strength (MPa)	Yield strength (0.2% offset; MPa)	Elongation (%)	Reduction of area (%)
CP-Ti Grade 4	550	485	15	25
CP-Ti Grade 3	450	380	18	30
CP-Ti Grade 2	345	275	20	30
CP-Ti Grade 1	240	170	24	30

According to the pureness and the processing elements like Fe, C, O, N, and H, pure titanium is available in four grades, as presented in Table 2 (John Nicholson, 2020).

**Table 2:** Constituents of pure titanium (CP–Ti) grades 1–4 (Jorge et al., 2013).

Components (%)		Fe max.	C max.	O max.	N max	H max.	∑	Ti (%)
ASTM grades	1	0.2	0.1	0.18	0.03	0.015	0.525	99.47
	2	0.3	0.1	0.25	0.03	0.015	0.695	99.3
	3	0.3	0.1	0.35	0.05	0.015	0.855	99.13
	4	0.5	0.1	0.4	0.05	0.015	1.095	98.93

*Ti* - titanium, *H* - hydrogen, *N* - nitrogen, *O -* oxygen, *C -* carbon, *Fe -* iron.

## 3 Properties of Ti and Ti alloys

The essential quality of Ti as biocompatible material is that it does not cause an unfavorable reaction when used in services. It's also necessary to have superior mechanical qualities, osseointegration, excellent wear, and corrosion resistance.

### 3.1 Biocompatibility

Implants are considered exceptionally non-toxic and unlikely to originate inflammation or allergic reactions (Williams et al., 2008). According to the tissue reaction, implants are classified as “bio tolerant,” which shows distant osteogenesis (formation of bone with ancillary interaction to the material), “bio-inert,” which shows contact osteogenesis, and “bioactive,” which shows bonding osteogenesis. While implants are revealed to human tissues and fluids, the factors that affect biocompatibility are (i) thrombosis, which is linked to blood coagulation and platelet adhesion to the surface of implants, and (ii) fibrous tissue encapsulation of implants placed in soft tissues (Viteri et al., 2013). Figure 1 depicts some of the biological effects that may cause by Ti implants.

**Figure 1:** Biological effect of an implant.

### 3.2 Mechanical properties

Hardness, rigidity, stretching, and Young's modulus is the most important mechanical features that aid in material selection. A crack generated by a mechanical malfunction on an implant is biomechanical unsuitability (Viteri et al., 2013; Luo et al., 2020; Zhang et al., 2022). Dental appliances must withstand forces during mastication; dental alloys must meet minimum mechanical properties requirements. Mechanical properties (Yadav et al., 2022) of some of the significant Ti alloys employed in dental and surgical treatment are shown in Figure 2 (Sarraf et al., 2022).

**Figure 2:** Mechanical characteristics of numerous titanium alloys for dental implants (Sarraf et al., 2022).

#### 3.2.1 Strength

Because today's exercises consistently put significant mechanical pressure on bones and joints, the design of an embed should be as reliable as possible. Titanium's quality and unbending nature contrast with noble combinations commonly used in dentistry (Jiang et al., 2014). Titanium composites can be made by combining them with other metals, such as iron, vanadium, or aluminum, to change their mechanical characteristics (Morinaga et al., 2018).

#### 3.2.2 Flexibility

The embedded materials must be adaptable to maintain a strategic distance from the pressure-protecting bones; due to this trademark, implant adaptability is critical. Titanium is applied for low modulus use when beta alloyed (along with niobium and zirconium), and its thermal development coefficient is comparable to that of humanoid bone, reducing the risk of embed disappointment. A higher modulus is required when alpha-beta alloyed (as with Ti) is applied for uses (for example, bone plates) (Elias et al., 2019). Titanium implants are thought to have extraordinary adaptability than cobalt-chromium cast fastens, allowing them to connect with more resounding undermines or be used in situations where smaller implants are required, like on premolar teeth ( Sun et al., 2022).

#### 3.2.3 Density

Cp Ti's thickness (4.5 g/cm^3^) is a fraction of the thickness estimated for many other base metals. Titanium is lighter (around 56 percent thick) than treated steel but has twice the yielding quality and nearly doubles the extreme elasticity. This stimulates the highest weight proportion of any metal suitable for clinical use (Gosavi et al., 2013).

#### 3.2.4 Non-magnetic

Cp-Ti, like all-titanium compounds, is unappealing. The charge levels of ferromagnetic and non-ferromagnetic materials are different. In addition, Ti is not distinguished by the metal locator, interfering with other metals (Emsley et al., 2011). Patients with Ti implants can be securely investigated with MRI as Ti is non-ferromagnetic.

#### 3.2.5 Low thermal coefficient of expansion

The low, warm coefficient of development of Ti, as opposed to the more significant part of other metals, makes it suitable for earthenware or glass materials. It also effectively helps Ti adheres to metal-glass or metal-artistic seals (Gosavi et al., 2013).

#### 3.2.6 Low modulus of elasticity

The modulus of the flexibility of Ti is many times greater than that of smaller bone. The immenseness of the plan in the best possible circulation of mechanical pressure move is the property of Ti. The flexibility modulus of the combination is generally higher than that of Ti, which is about 5.6 times that of minimal bone (Philip et al., 2017).

### 3.3 Shape memory

In the shape memory alloy of Ti and Nickel, in 1968, Johnson and Alicandri introduced NiTi as an implant material (Castleman *et al.*, 1976). NiTinol, as a super-elastic or pseudo-elastic alloy, for biomedical applications, is made for orthopedic and orthodontic implants (DI *et al.*, 1996; Sharma et al., 2008). Again, Nitinol is used in endodontics to shape and clean root canals throughout root canal procedures. However, embedded materials are the main driver of clean titanium and Ti–6Al–4V composites. Lately, a form of Ti composite made of non-harmful components such as Sn, Mo, Zr, Ta, Nb, or with a lower module of flexibility and higher quality, has grown (Kurod et al., 1998).

### 3.4 Chemical properties

In the oral cavity, significant variations in pH and temperature occur regularly. Dampness, corrosive conditions, and antacid or other compound operators may all degrade the stuff. Different materials such as water, oxygen, chloride, and sulfur are available that cause mechanical dissatisfaction in dental compounds due to ingestion, significantly affecting the material's durability and consistency (Iijima et al., 2010). Water-synthesized Ti has the greatest biocompatibility of all metals. No matter how you look at it, the research on the consequence of toxins and surface medicines of Ti implants on bony joining was groundbreaking (Bhola et al., 2010). Because of its warmth sensitivity, Ti has a typically negative reversible ability). Ti and Ti combinations can change effectively, prompting unconstrained re-passivation regardless of whether the obstruction layer gets disturbed (Koijumi et al., 2019; Alkhadashi et al., 2020).

Regarding dental implant methods (implant fixings and abutments) and prostheses (dental metal-ceramic crowns and changeable denture frameworks), Ti and its alloys have long been the preferred materials. After coming into contact with the surrounding environment, Ti has extremely high resistance to corrosion in physiological solutions. The Ti also has outstanding biocompatibility due to the development of defensive titanium oxide (TiO_2_) film on the metal surface when interacting with the external surroundings (Souza et al., 2015).

### 3.5 Wear behavior

Wear is common at the junction of counterfeit joints. Between the embed and the bone meddle, the lower layer of the bone undergoes a change cycle that causes osteolysis. Titanium's superior corrosion confrontation, overall biocompatibility, and low Young's modulus comparable to traditional hardened steels and cobalt-based composites make it an excellent choice for biomedical uses (Ding et al., 2018; Revathi et al., 2017). Extraction of restorative Ti surfaces can occur during the chewing process due to frictional surface contact with opposing surfaces, hard particles initiated from nutritional sources, food bolus, toothbrushes, and paste (Lambrechts et al., 2006).

Munching friction on Ti can erode the TiO_2_ coating, resulting in material loss and probable failure of dental implants and prostheses. Metallic ions are generated due to wear and corrosion processes, and particles instigating from Ti have been identified in the adjacent tissues and linked to inflammatory processes. As seen in Figure 3, various tribocorrosion processes can occur during contact between ductile metallic Ti and a strong inert counter-body (alumina). (Souza et al., 2015).

**Figure 3:** Tribocorrosion processes of Ti implants (Souza et al., 2015).

### 3.6 Osseointegration

At all stages of bone recovery around oral Ti inserts, irritation, recovery, and redesigning occur with a conceivable cover. Both mending types show a minor departure from the cell and sub-atomic level in the absence of proximity of Ti implants. The Ti implant surface affects the underlying arrangements of protein adsorption, platelet grip, hemostasis, aggravation, and osteogenic cell reaction (Tan et al., 2006; Elias et al., 2010). One of the primary initial phases in the cell reaction to a biomaterial is cell connection to the implant's surface. Attachment receptors, such as integrin, mediate the cell-cell connection through a protein-rich layer. When an implant is precisely positioned inside the bone, several natural, physical, synthetic, warm, and other factors influence whether osseointegration occurs.

The timetable for osseointegration of dental implants is depicted in Figure 4. Within four weeks, the development of new bone is noticeable on the implant's surface, which connects with bone that has already developed on the host bone (distant osteogenesis). At some point between 8 and 12 weeks, the peri-implant boundary is entirely substituted by mature lamellar bone in direct connection with the implant surface, bringing osseointegration to an end (Wang et al., 2015).

**Figure 4:** Osseointegration Timeline of dental implants (Wang et al., 2015).

Due to its outstanding biocompatibility, high quality, and break sturdiness, Ti, and its compounds have been widely applied for dental and orthopedic implants under load-bearing circumstances *(*Li et al., 2020). Despite direct clinging to the bone, they don't produce a synthetic bond with bone tissue (Figure 5(a-b)). However, despite its excellent biocompatibility, the hydroxyapatite covering has a few drawbacks, including delamination of the covering layer from the substrate, challenges in regulating the structure of the covering layer, and debasement of the covering layer itself, which can result in garbage becoming a wellspring of third body degradation (Liu et al., 2005). By using appropriate embed surface medicines, electrochemical testimony, plunging, and physical fume statement methods, steady bone tissue can achieve a stable and robust issue that remains to be worked out in association with the bone-embed interface (Kim et al., 1996). Ti–6Al–4V implants, with medical success rates of up to 99% at ten years, have been used to fabricate dental implants since around 1981 are biocompatible with bone and the gingival tissues and are experiencing osseointegration (John Nicholson, 2020).

**Figure 5:** (a) TEM images of osseointegration of dental implants b) SEM image of the bone-implant interface after 3-week (James et al., 2017).

### 3.7 Surface characteristics and wettability

Appropriate surface roughness promotes interfacial adhesion and decreases the chance of ionic leak and peri-implantitis. 1–2 mm of roughness may be used to establish the stability of these two characteristics. External topographies have been widely studied to determine their influence on Osseointegration and the functional integrity of dental implants. The impact of surface quality on gene regulation and neighboring skeletal surface reactions is critical in implant quality. As a result, enhancing the implant surface roughness with Nano roughness is required to give numerous bonding locations for cell amalgamation, resulting in effectiveness and facilitating high-speed Osseointegration (Wennerberg et al., 2009; Albrektsson et al., 2016; Salerno et al., 2015; Kandavalli et al., 2021).

Surfaces with a wetting tension >30 mN/m are hydrophobic, while those below 30 mN/m are hydrophilic (Gittens et al., 2014). A hydrophilic surface with a water contact angle of 40–70 is excellent for bio-response among human body fluids and cells (Wang et al., 2020). The dental implant volume affects the implant's biogenesis when the contact angle is changed. It also increases contact with biological substances and cells (Gittens et al., 2014). Dental implants with extremely hydrophilic and irregular surface interfaces are still the best candidates for osseointegration (Sawase et al., 2008). Hydrophilic surfaces are preferred over hydrophobic surfaces due to their affinity for cells and biological substances. Chemically treated Ti surfaces with increased hydrophilicity and surface-free energy can abridge hydrocarbon contamination (Rupp et al., 2006; Elias et al., 2008).

### 3.8 Antibacterial property

Infections induced by microbes that are introduced by the implant are key contributors to the failure of implants. Since it begins immediately after bacterial adherence, the creation of biofilm is the primary cause of infections. Once a biofilm has formed on an implant, it is tough to eradicate any germs that may have colonized there. Therefore, the antibacterial qualities of the implant play a significant role in ensuring the implant's success over a long period. Coatings made of silver (Ag), coatings implanted with fluoride (F) or chloride (Cl), coatings made of titanium nitride (TiN), coatings made of hydroxyapatite, coatings made of Hyaluronic acid, and coatings made of titanium dioxide (TiO_2_) all exhibited potent antibacterial activity (Esteves et al., 2022; Parfenova et al., 2022).

## 4 Manufacturing of Ti and Ti alloy dental implants

### 4.1 Casting

Titanium has a greater melting point than traditional dental metals, and high-temperature melting processes, like arc melting, are required. Furthermore, as titanium oxidizes easily at high temperatures, ambient gases must remain inert during melting and casting. Even the mold's oxide component should have been resistant to molten titanium. Furthermore, new techniques were required to provide acceptable casting pressure due to titanium's low density. As a result, entirely new dental casting equipment with Ti was required. The production of a partial denture employing Ti casting in the United States was described in 1978 (Waterstrat et al.,1978). An arc melting pressure casting equipment with an argon environment was invented in Japan, and to generate the required casting pressure, vacuum pressure or centrifugation was developed ((Hamanaka et al., 1989; Ida et al., 1982). The reports on the castability of Ti and Ti-alloys are summarized in Table 3.

**Table 3:** Research of the Ti cast-ability (Koizumi et al., 2019).

Casting Machine	Investment material	Casting metal	Ref
Centrifugal casting machine	MgO	Ti–6Al–7Nb, Ti–15Mo–5Zr–3Al, CP-Ti	(Koizumi et al., 2018)
	MgO, Al_2_O_3_ + MgO	CP-Ti	(Reza et al., 2010)
	MgO	Ni–Cr, Au alloy, CP-Ti	(Watanabe et al., 2000)
Argon gas pressure casting machine	SiO_2_	Co–Cr, Ti–6Al–7Nb, CP-Ti	(Wang et al., 1999)
	SiO_2_, ZrSiO_4_	CP-Ti	(Takahashi et al., 1993)
	MgO, SiO_2_	Ti–6Al–4V, CP Ti, etc.	(Ida et al., 1982)

Titanium is very responsive at high temperatures and easily responds to oxygen. As a result, it reacts with oxides like silica (SiO_2_), the major constituent of most investment casting materials. The Ti investment casting material must maintain its reliability at high melting temperatures, be chemically constant, not oxidize Ti, and exhibit casting shrinkage-compensating qualities. Steady oxides such as zirconia (ZrO_2_), magnesia (MgO), and alumina (Al_2_O_3_) were researched as refractory ingredients as a replacement for SiO_2_ to produce investment materials that fit such characteristics (Kudoh et al., 1996). When it came to combining the best casting machinery with the best casting venture materials, the radial projecting apparatus combined with MgO-based speculation materials free of phosphate produced excellent Ti castability (Ida et al., 1982; Reza et al., 2010).

A Ti casting framework (Figure 6 (a-c)) can also be utilized for more durable dental prostheses. Mechanical characteristics of Ti–6Al–7Nb composite have been reported to be of sufficient quality and lengthening: Tensile quality was rough twice that of Ti and only a few percent lower than that of the Ti–6Al–4V compound. Simultaneously, it stretched nearly 40% more than the Ti–6Al–4V combination (Pieralini et al., 2010). The Ti–6Al–7Nb amalgam consumption resistance was investigated using long-distance inundation and anodic polarisation techniques, and it was discovered that this composite would be preferable to the Ti–6Al–4V compound, which was comparable to Ti in terms of erosion resistance (Rodrigues et al., 2012). With fewer casting imperfections than a one-chamber vacuum projecting framework designed for Ti, the liquid Ti–6Al–7Nb mixture progressed almost identically to pure Ti and better than cobalt-chromium amalgam (Srimaneepong et al., 2005; Wang et al., 1999).

**Figure 6:** (a) Ti framework; (b) Clinical fit over the implant abutments; (c) Installed prosthesis (Silveira et al., 2012).

### 4.2 Additive Manufacturing/3D printing of Ti dental implants

In metal powder-based added substance manufacturing methods, various parts are delivered by softening metal powder layer by layer under the influence of an electron or a laser (Fang et al., 2017). The 3-dimensional (3D) CAD (computer-aided design) model is the starting point for Additive Manufacturing innovations, which can be created in a CAD framework or acquired through research, such as 3D scanners or PC tomography. Figure 7 shows a schematic demonstrating the design and manufacturing procedure of a patient-distinctive mandibular prosthetic device for maxillofacial restoration.

**Figure 7:** Design and production of a patient-distinctive mandibular prosthetic implant (Sarraf et al., 2022).

Additive Manufacturing techniques produce tissue, organs, prosthetics, implants, and anatomical models. Powder-based cycles, such as laser powder bed combination (LPBF), also known as selective laser melting (SLM) and Electron Beam Melting (EBM) and coordinated vitality testimony (Directed Energy Deposition (DED), for example, Laser metal deposition (LMD), are progressively being used in various biomedical sectors (Trevisan et al., 2017). Some of the dental prostheses manufactured by 3DP/AM are shown in Table 4. Also, Figures 8 and 9 illustrate Ti frameworks for the edentulous jaw.

**Table 4:** Ti and Ti alloys dental prosthesis depending on various 3DP/AM fabrication systems (Revilla et al., 2020; Huang et al., 2022).

3DP/AM Techniques	Applications	Significant Findings	References
Selective Laser Melting (SLM)	Dental Implant	Superficial roughness (Ra) (SLM): 10.65 ± 2.3 μm Water contact angle: 86.97 ± 2.65°	Shaoki et al., 2016
	Surgical guides and implants in bimaxillary orthognathic surgery	High Accuracy left-right (0.3 mm), up-down (0.33 mm), and anterior-posterior positioning (0.7mm)	(Heufelder et al., 2017)
Electron Beam Melting (EBM)	Root Analog	Micro porosities characteristics of the specimens stimulated bone in growth and improved bone bonding.	(Ramakrishnaiah et al., 2017)
	Cutting guides and fixation plates in bimaxillary orthognathic surgery	Post-operative nerve parenthesis was recovered within 2–3 months Achieve good final occlusion.	(Li et al., 2017)
Direct Metal Laser Sintering (DMLS)	Immediate dental implant in the anterior maxilla	Efficient aesthetic integration (1-year follow-up)	(Figliuzzi et al., 2019)
	Immediate dental implant	100% survival rate (1-year follow-up)	(Mangano et al., 2014)
Direct Laser Metal Fusion (DLMF)	Root Analog	The specimen was clinically steady with no contamination,	Figliuzzi et al., 2012)
	Dental implant	94.3% success rate and 94.5% survival rate (3-year follow-up)	(Tunchel et al., 2016)

**Figure 8:** Laser-welded Ti framework (Örtorp et al., 1999).

**Figure 9:** Ti-metal framework for implant-supported prostheses (Revilla et al., 2020).

Uncoated standards embed fatigue resistance increases by 1/3 compared to coated implants made with 3D printing (Gruner et al., 2001). Co-sintering forerunner particles, powder plasma splashing over a high-thickness center, Ti strands sintering, and stable state foaming by extension of argon-filled pores are some of the techniques that have been proposed for obtaining porous Ti structures (Li et al., 2006). Late 3D printing/added substance fabricating (3DP/AM) innovations can now comprehend Ti platforms, giving them unlimited control over the outside shape math and the interconnected pore system (Traini et al., 2008).

Diverse in vitro studies have inspected the cell reaction to the outside of AM/3DP implants after watching the development of the human fibrin cluster and the actions of human mesenchymal foundational microorganisms and human osteoblasts (Mangano et al., 2009, 2010, 2011). Furthermore, numerous animal studies (Alkhadashi et al., 2020) and humans (Jiang et al., 2014) have documented the bone reaction to 3DP/AM Ti implants. In addition, more than some animals and humans have archived histological morphometrics about the bone reaction after AM/3DP Ti implants (Witek et al., 2012; Stubinger et al., 2013; Mangano et al., 2013; Shibli et al., 2013).

3DP/AM, the most attractive methods for the production of implants: (i) swiftness, (ii) precisely controlled the requirement of the patient, (iii) exact shape and dimension, (iv) quality of different living tissues, (v), especially on techniques and procedures, and (vi) effectual variables for porous scaffolds, density, taking pore size, etc., into concern. It is postulated that 3DP is becoming a popular method for Ti, Ti6Al4V, shape memory alloys, and cobalt-chromium alloys. AM implants would comply with custom-built designs, rapid production, biocompatibility, suitable strength, elastic modulus, surface conditions, etc. (Attarilar et al., 2021).

Ti–6Al–4V implants have excellent biological and mechanical properties for applications because failure rates over substantial periods are meager and survive for over ten years. Therefore, it is plausible that CAD/CAM-based 3D printing could make these implants more effective for the critical development of osseointegration of releasing bone cells (20–50 nm) which initiates the steps that result in bone formation (John Nicholson, 2020).

The yield strength, tensile strength, and hardness values were compared under the Ti alloy Ti-64 for 3D printing (SLM) and metallurgical process (static tests). Mechanical properties are higher for additive manufacturing than conventional methods (rolled bars). Table 5 lists some of the significant properties that 3D printing can achieve after advancements:

**Table 5:** Comparison of Mechanical properties obtained for Ti-64 received by 3D printing and metallurgical methods (Karolewska and Liga, 2019; Quintana and Tong, 2017; Rehounek et al., 2018; Kim et al., 2020).

Fabrication Methods	Yield Strength (S_y0,2_, MPa)	Tensile Strength (S_u_, MPa)	Hardness (H, GPa)	Tensile Strain (%)	Flexural Strength (MPa)	Flexural Modulus (GPa)
3D printing (SLM)	1225.7	1360	5.19	12.33	2200	40
Metallurgical method	1107	1126	4.58	-	-	-
Cast Ti	-	-	-	5.88	-	-

A comparison of surface characteristics of Additive Manufactured (AM) samples and other surface-modified samples (AM + sand-blasted and AM + polished). SEM image confirmed that the Additive Manufactured sample contained spherical particles (unsintered powder) on the surface, but surface treatment (AM + sand-blasted and AM + polished) removed the unsintered spherical particles. The surface roughness (Ra) from the measurements is shown in Table 6 below (Kim et al., 2020).

**Table 6:** Surface roughness of additive manufactured Ti alloy.

Specimens	Surface roughness (μm)
AM specimen	8.3 ± 0.2
AM + sand-blasted	2.3 ± 0.3
AM + polished	0.6 ± 0.1

## 5 Surface modification of Ti implants

Topology and surface geography is critical for achieving dental implants' short- and long-term benefits (Guéhennec et al., 2007; Lee et al., 2014). Surface treatment improves wettability and thus (Nakae et al., 2005) enhances bone connection with the surface of dental implants. Adequate cell adhesion, proliferation, and accelerated osseointegration are required for an implant to succeed (Sollazzo et al., 2008).

### 5.1 Surface roughening

The surface roughness of dental inserts influences the rate of osseointegration and biomechanical fixation, according to a study by Brett et al. who discovered that the quality articulation of osteoblast cells augmented with an escalation in surface roughness (Brett et al., 2004). These qualities were dubbed harshness. Surface roughness is separated into three levels based on the size of highlights: large-scale, micro, and nano-sized topologies (Guéhennec et al., 2007). Geographical highlights in millimeters to many microns are acquired at the Macro level. In this case, high harshness promotes early mending and obsession and long-term mechanical security; however, it increases the risk of periimplantitis and ionic spillage (Becker et al., 2000). The micro topographic profile of inserts for surface alteration ranges from 1-10 m, but the ideal surface should theoretically be bonded with hemispheric destruction around 1.5 m top bottom and 4 m in diameter (Hansson et al., 1999). Geology in the nanometer ranges is essential for protein adsorption, osteoblastic cell attachment, and osseointegration speed (Brett et al., 2004).

Roughening dental implant surfaces can be done by various methods (Shayganpour et al., 2015; Muthaiah et al., 2022). Roughness sizes vary depending on the surface treatment. The topography and characteristics of implant surfaces had a role in osseointegration and the long-term survivability of dental implants. Numerous surface treatment approaches of diverse dental implant schemes are summarized in Table 7, and Figure 10 (a-d) compares the SEM images of some of the treated Ti surfaces (Rimal U et al., 2018).

**Table 7:** Numerous surface modification approaches for dental implant systems (Rimal U et al., 2018).

Surface Treatment	Materials and method	Special Feature	Reference
Ablative Procedure			
**Acid Etching:** Etching with strong acids which produces micro pits of 0.5–2 μm	HCL, HNO_3_, HF, H_2_SO_4_	By forming Ti hydride, Escalate the hydrogen concentration	(Degidi et al., 2003; Iwaya et al., 2008)
**Anodizing:** titanium oxide layer is roughened by the electrochemical cycle	Strong acids (HF, H_3_PO, HNO_3_, H_2_SO_4_) are utilized for galvanostatic-anodization of Ti surface at high current density (200A/m^2^) or potential (100 V).	Oxide thickness: between 600 and 1000 nm.	(Sul et al., 2001) (Marenzi et al., 2019)
**Grit Blasting:** Pressurized Particles are projected onto the implant surface by Nozzle	Hydroxyapatite (HA), Aluminum dioxide, and Titanium dioxide	Further acid etching is required.	(Shemtov-Yona et al., 2014)
**Laser Treatment:** Can be used to change the surface of an implant for osseointegration or to treat periimplantitis.	High-power laser strikes on the defensive layer that covers the metallic surface.	The embed shows a honeycomb design with tiny pores	(Berardi et al., 2008)
**Additive Procedures**			
**Plasma-spraying:** Used to lay down a thick layer of coating materials.	Thermal spraying of Ti and Hydroxyapatite	A film thickness of a few millimeters to a few micrometers is formed	(Ong et al., 2004)
**Electrophoretic Deposition of Hydroxyapatite:** HA is an osteoconductive material that can frame a reliable connection between the bone and the embed.	It consists of two steps: the dispersion of charged particles in a liquid solvent under the influence of a functional electric field (electrophoresis), and the congealing of particles to create an adherent layer on the electrode (deposition)	The coating obtained by this technique is finally sintered at 800 °C.	(Meng et al., 2008)
**Sputter Deposition:** A robust methodology in taking out material-property discontinuities to build grip quality is by evaluating the material synthesis close to the interfaces or through the coatings.	Radiofrequency magnetron sputtering methods	Significantly increase adhesion strength	(Ding, 2003)
**Sol-Gel Coating:** Ti implants are immersed into the gel and quickly hermos-cycled at 600 °C	The precursor is typically produced in ethanol at the sol stage before being thermally cycled into a gel with a specified viscosity.	Several coatings and thermos cycling is required to attain the preferred thickness of the coat.	(Jaafar et al., 2020)
**Biomimetic Precipitation:** This procedure considers the nucleation and development of bone-like precious stones on a pretreated substrate	Calcium phosphate under physiological conditions (37 °C and pH = 7.4).	This strategy can be altered for the fuse of medications or development features onto the embed surface along these lines making the inserts osteoinductive and osteoconductive.	(Kreller et al., 2021)

**Figure 10:** Surface morphology of Treated Ti surface (a) sandblasted and etched with warm HCl (Kim et al., 2008); (b) Plasma sprayed (Jemat et al., 2015); (c) Anodized (Elias, 2011); (d) Sol-gel coating (Jaafar et al., 2020).

### 5.2 Chemical, electrochemical, and thermal modifications

A few trial results on substance, electrochemical, warm, and blends for modifying the Ti surface to improve surface compound, mechanical, and natural responses. Endo-treated NiTi in 30% NHO_3_, which was then heated at 400 °C for 0.75 h before the NHO_3_ treatment, followed by boiling in water for 6–14 h (Endo et al., 1995). The treated NiTi surfaces were tested for disintegration resistance in cow-like serum. It was discovered that (i) Because of stable rutile oxide (TiO_2_) development, those stems that were thermally treated had significantly lower metal particle discharge, and (ii) Glutaraldehyde was used to covalently immobilize human plasma fibronectin (a glue protein) onto an alkylaminosilane derivate of NiTi substrate and (iii) According to the XPS spectra, gamma-aminopropyltriethoxysilane (-APS) was clung to the surface via metallosiloxane securities (Ti–O–Si) framed using a buildup response between the silanol end of -APS and the outside of the hydroxyl gathering, with an exceptionally cross-connected siloxane arrange shaped after warming the silanized surface to 100 °C. Given these findings, it was hypothesized that human plasma fibronectin was immobilized in the body, promoting fibroblast spreading; suggesting that this concoction change could be a compelling method for controlling metal/cell associations (Endo et al., 1995; Krozer et al., 1999). CPTi was first impacted with 354–500 m enormous cornmeal in a study done by Rupp et al. (Krozer et al., 1999), followed by (1) HNO_3_/HF/HCl scratching, (2) H_2_SO_4_l/HC drawing, (3) HF/H_2_SO_4_/HCl/oxalic corrosive + killed, and (4) HF/H_2_SO_4_/HCl/oxalic corrosive (Macdonald et al., 2004) The microstructure, compound arrangement, and wettability of thermally and artificially adjusted Ti–6Al–4V circles were investigated, and the results were linked to the level of adsorption between radiolabeled fibronectin and the Ti–6Al–4V combination surface, as well as the subsequent bond of osteoblast-like cells. After water and hydrogen plasma drenching particle implantation (PI3) (Xie et al., 2005, Rohanizadeh et al., 2004), the surface bioactivity of titanium was investigated.

## 6 Applications of Ti and Ti alloys in dentistry

Recently, titanium has sparked much attention in dentistry. Since its outstanding resistance to corrosion, biocompatibility, and favorable mechanical and physical qualities, titanium (Ti) uses in dentistry (Figure 11) have increased considerably in recent years. Some of the commonly used Titanium alloys and their properties are shown in Table 8.

**Figure 11:** Titanium and Ti Alloys in dentistry.

**Table 8:** Properties of Ti alloys (Osman et al., 2015).

Material	Modulus (GPa)	Ultimate Tensile Strength (MPa)	Yield Strength (MPa)	Elongation (%)	Density (g/cc)	Type of Alloy
Ti–6Al–4V- ELI	113	860	795	10	4.4	α + β
Ti–6Al–4V	113	930	860	10	4.4	α + β
Ti–6Al–7Nb	114	900–1050	880–950	8–15	4.4	α + β
Ti–5Al-2.5Fe	112	1020	895	15	4.4	α + β
Ti–15Zr–4Nb–2Ta-0.2Pd	94–99	715–919	693–806	18–28	4.4	α + β
Ti–29Nb–13Ta-4.6Zr	80	911	864	13.2	4.4	β

### 6.1 Titanium in dental implants

Dental implants are frequently utilized to support prostheses and supplant missing teeth. Figure 12 shows an exceptional fitting between a Ti-based abutment (de Holanda Cavalcanti Pereira et al., 2022) and an implant that has adequate mechanical strength and masticatory force distribution in an implant-supported prosthesis (Souza et al., 2015). As shown in Figure 13, endosseous implants may be used in the invaded jaw and splint with a screw-retained full-arch renovation. Modern implants are frequently designed with a screw thread by which the components are fixed with the mandible or maxilla bone (Baumgarten, 2018).

**Figure 12:** Titanium-based abutment-implant joint (Souza et al., 2015).

**Figure 13:** Endosseous titanium implant for hybrid restoration of Maxillary and mandibular (Baumgarten, 2018).

### 6.2 Titanium in restorative dentistry

Dental restoration (Figure 14) replaces or repairs damaged teeth lost due to decay or injury. Restorations on individual teeth are often filled with filler materials to cure decay. More wide-ranging refurbishments, such as dental bridges, crowns, and implant-aided restorations, are also done with patient-specific restoration techniques ((Baumgarten, 2018; Močnik and Kosec, 2021).

**Figure 14:** Titanium in restorative dentistry a) Filling of Dental decay, b) Ti crown covered with porcelain c) Spatula (Philip et al., 2017).

Due to its unattractive appearance, Ti and its alloys are rarely employed for treating decay. However, because of their excellent durability and affordable price, dental restoration with titanium crowns is an option many individuals opt for. An alloy of nickel, chrome, and titanium with 4%–6% titanium makes up the inner structure of a titanium crown, which has an outer shell composed of Ceramco3 porcelain. The mouth's saliva does not affect the crown, nor does the oral environment cause it to oxidize. This is the greatest option, especially for those with severe metal allergies (Haag, 2011).

Moreover, Dental composite filling instruments (spatula) are often made with Ti alloy or coated with Ti alloy. For composite resins and glass ionomers, TiN-coated stainless steel instruments produced no decrease in adhesion compared to non-coated, clean, polished stainless steel instruments (Philip et al., 2017).

### 6.3 Orthodontic applications

Orthodontic braces are affixed to the teeth, and orthodontic wiring is threaded through the bracket and ligated to hold it in place. Recently, orthodontics (Figure 15) has extensively used temporary anchorage devices (TADs). Most of these devices are embedded in the patients' bone/soft tissues, so they should be biologically compatible. Most of the TADs are made of titanium alloys. They have been used as anchorage devices to move teeth in directions that generally are difficult to move without additional conventional anchorage methods. Although Stainless steel has been used as cheaper TADs than titanium-based TADs, Titanium still provides superior properties to Stainless steel TADs (Rokaya et al., 2021).

**Figure 15:** Orthodontic applications.

### 6.4 Endodontic applications

Endodontic therapy entails removing contaminated tissue from a tooth’s root canal system, contouring and disinfecting the canals, and refilling the canals with the appropriate ingredients. In endodontics, using rotary files (Figure 16) made of nickel-titanium (NiTi) has revolutionized root canal treatment (Dobrzański et al., 2022).

**Figure 16:** Endodontic application of Rotary file (Philip et al., 2017).

### 6.5 Maxillofacial and oral surgery applications

Oral and maxillofacial surgical treatment includes temporomandibular joint, bone grafting, orthognathic, dent alveolar, and correcting the face's fractures and soft tissue deformities. Titanium and its alloys significantly contribute to each of these fields. Many of these treatments necessitate an implanted maneuver to either exchange or stabilize a lost portion or sections, allowing for smooth healing. Because Ti appears clinically inactive, producing little or no tissue inflammation, it has primarily replaced stainless steel and Vitallium in maxillofacial and oral surgery.

Figure 17 (a) shows a Ti–6Al–4V arch bar fastened into both the maxilla and mandible used to alleviate the jaws after the restoration of a mandibular rupture (IIzuka et al., 2006). Maintaining space under the soft tissue for the extra volume of the placed graft is crucial when bone grafting is essential to enlarge the size of the bone. Figure 17 (b) shows that Ti mesh is frequently employed to keep the distance between a particulate xenograft and a deficient maxilla (De Angelis et al., 2015).

**Figure 17:** (a) Repair of mandibular fracture. (b) A particulate xenograft is used to enhance a defective maxilla (Baumgarten, 2018).

## 7 Limitations of Ti and Ti alloys as dental implants

Implants made by Ti have an extensive track of expectable medical outcomes, with a total accomplishment rate of 98.8% for a long time (Lindquist et al., 1996). This can be attributed to CpTi and Ti–6Al–4V's great biocompatibility, significant bone, mild tissue reaction, and satisfactory quality and consumption obstruction. Recently, there has been progress in searching for replacements for Ti–6Al–4V and CpTi to counteract a few disadvantages of Ti dental implants. Those drawbacks can be grouped into stylish tests, medical issues, and progress in bio-artistic events. Test of taste: Patients can benefit from improved modern reproduction because fired materials are white and imitate natural teeth better than dark Ti. When the delicate mucosa is of thin biotype or retreats after some time, using white artistic implants would block Ti implants' dim shine (Den et al., 2008; Cosyn et al., 2012). In writing, the expansion of keratinized tissue around inserts is accounted for using autografting with subepithelial connective tissue or xenogeneic collagen framework of porcine root (Schneider et al., 2011; Esposito et al., 2012). However, there is no concrete evidence that joining thin tissue thickens it. Medicinal issues: Ti is not currently considered an entirely bioinert material; rather, it may be an allergen, as evidenced by a few studies (Evrard et al., 2010; Pigatto et al., 2009). Raised concerned with Ti alloys have been discovered in the region of oral inserts (Koutayas et al., 2009), pee (Jacobs et al., 1998), serum, and local lymph hubs (Onodera et al., 1993), all of which are potentially harmful to the human body. In any case, the clinical relevance of the above discoveries is unclear, as various studies have previously confirmed Titanium's dependability for long-term usage in the oral circumstance (Wenz et al., 2008). These phenomena, combined with the aesthetic matter, have led some dental patients who are mentally fearful of demanding treatment with metal-free dental implants.

## 8 Recent advances in Ti-based implant materials

Several examples in titanium-based biomaterials ' imaginative work demonstrate the ability to make mixes made of no allergenic and nontoxic segments with inspiring mechanical characteristics (low modulus and high caliber) and workability. Other non-toxic ingredients, like Zr, Pd, Nb, Ta, Mo, and Fe, are being developed to replace vanadium and aluminum in future developments (Niinomi et al., 2003). These are composites with a lower modulus of flexibility (55–85 GPa), similar to bone (17–28 GPa). This lower adaptability modulus is appealing because it allows for more precise weight movement at the bone-installation interface. Additionally, these composites are designed to achieve higher caliber and quality than ᾳ + β mixes. Another compound (Roxolid®, Straumann, and Basel, Switzerland) for collecting slight separation across embeds has recently been introduced to dentistry. The foundation is the blend's two-part itemization of 83–87% Ti and 13–17% zirconium. With a 953 MPa inflexibility rating and 40% higher weariness strength than Ti–6Al–4V and CpTi, this composite has been determined to have superior mechanical properties (Grandin et al., 2015). When zirconia is added to Ti, osseointegration improves, and the combined material is more biocompatible than pure Ti (Bernhard et al., 2009). Ti-12.5Zr-2.5Nb-2.5Ta is another good Ti mixture for careful installation (TZNT). When compared to standard Ti mixes, this composite had an exclusive benefit in that its modulus of flexibility was closer to that of human bone (100 Gpa–120 Gpa) and had a nearly identical affirmation strain (0.65%) as human bones (0.67%) (Ikarashi et al., 2005). The addition of Zr, Nb, and Ta to the compound, for example, has shown no adverse tissue reactions or toxicity and has a high resistance to disintegration (Li et al., 2003, 2004).

## 9 Futuristic development of innovative dental implants

The Ti–6Al–4V compound is a better substitute for CPTi because it has better mechanical and consumption resistance and a lower flexibility modulus (Long et al., 1998). However, numerous attempts have been made to enhance its characteristics, particularly those associated with versatile modulus, consumption obstruction, and biocompatibility. Furthermore, there have been reports that aluminum and vanadium particles can cause neurological issues like Alzheimer's disease and unfriendly tissue responses over a long period (Brunette et al., 2001). Hence, there is a pressing need to create new Ti amalgams, primarily by adding non-cytotoxic components such as niobium, molybdenum, tantalum, and zirconium. Parallel composite Zr–Ti is the most promising. Both in vitro (Eisenbarth et al., 2004) and in vivo (Saldana et al., 2007) evaluations have shown that zirconium as an endosseous embed has excellent biocompatibility. Regardless of the certainty of metal particle discharge throughout biocorrosion, the harmfulness of Zr particles is recognized to be negligible due to the deficiency of biomolecule blend (Hanawa et al., 2004). Zr is synthetically similar to Ti; when added to a firm arrangement with Ti, it is considered an unbiased component because it has an indistinguishable allotropic change and a comparable stage progress temperature. Prior research has shown that combining zirconium with robust arrangements can reduce the martensitic change temperature of Ti (Ho et al., 2008). Titanium's liquefying temperature can also be reduced by expanding zirconium, lowering projecting and swaging costs (Ho et al., 2009). Because of the vast temperature dissimilarity between the liquid composite and a much more excellent venture, lowering Titanium's liquefying temperature could reduce its interaction with oxygen and decrease the possibility of defective filling and resulting porosity improvement (Eboungabeka et al., 2021). Correa et al. (2014) recently looked into the biocompatibility, mechanical characteristics, and microstructure of Ti–Zr alloys containing 15, 10, and 5% zirconium. They discovered that Ti–Zr alloys are primarily composed of the α-phase (with hcp arrangement) and have significantly higher miniature hardness values than CPTi. The versatility modulus of the composites was sensitive to zirconium fixations while remaining within the range of regular Ti amalgams (Correa et al., 2014), and the amalgams had no cytotoxic possessions on osteoblastic cells under the conditions examined.

Ti–Zr–Nb–Ta (TZNT) is another promising dental implant combination (Nag et al., 2009). Quaternary Ti alloys are considered superior to business ternary (Samuel et al., 2010) and twofold composites in erosion resistance (Karthega et al., 2007). Metals such as Zr, Ta, and Nb have also been excellent biocompatibility and osteoconductivity (Payer et al., 2010; Rosalbino et al., 2011), with no known adverse effects on humans. The Ti–Nb–Zr–Ta composites were found to have similar cell multiplication but greater cell separation than the Ti–6Al–4V composites (Samuel et al., 2010). In comparison to Ti, Ti–20Nb–10Zr–5Ta (TNZT) has improved inactivity, hardness, and extreme rigidity (883 MPa), as well as a lower versatile modulus (59 GPa) (Milosev et al., 2013; Popa et al., 2012). Furthermore, this alloy appeared to have no adverse situation on cell endurance, apoptosis acceptance, development interruption, or antacid phosphatase movement compared to Ti, indicating that Ti–20Nb–10Zr–5Ta in dental applications is feasible (Milosev et al., 2014).

## 10 Futuristic surface modification of Ti-based dental implants

Recent surveys have proposed a few procedures (Bauer et al., 2013) to improve the speed and quality of osseointegration of Ti implants. These future patterns concern (1) Surface roughness can be adjusted at the nanoscale to improve protein adsorption and cell grip (Zhang et al., 2013), (2) biomimetic calcium phosphate coatings for improving osteoconduction (Shadanbaz et al., 2012), (3) combining natural medications to speed up the bone remedial progression in the peri-embed area (Choo et al., 2013; Zhang et al.,2014) and (4) natural segments with nanoparticles (Qiao et al., 2015; Memarzadeh et al., 2015), Chlorhexidine and polysaccharides are two examples, with chitosan receiving special attention (Wang et al., 2004, 2006; Scharnweber et al., 2007). A technique of current interest is Nano topographical alterations on the embed surface to persuade inherent osteoinductive motioning of the surface follower cells. Existing evidence for Nano topography suggests that basic osseointegration steps can be regulated by nanoscale changes in the embed surface (Puckett et al., 2008; Park et al., 2009; McNamara et al., 2010). The embed's surface collaboration with particles and proteins is altered due to these changes (i.e., adsorption, arrangement, bioactivity, etc.). These connections can greatly impact subatomic and cell exercises and the osseointegration cycle. Endosseous inserts are altered Nano topographically using various strategies and approaches (Subramanian et al., 2012). Physical techniques for compaction of nanoparticles to produce surfaces with nanoscale grain limits (Webster and Ejiofor, 2004), Chemical Treatment (Cooper et al., 2006), creative sandblasting/acid etching (Ellingsen et al., 2006), optical lithography (Domanski et *al.*, 2012), galvanostatic anodization (Sul et al., 2005), and crystal deposition (Lee et al., 2006, 2012). Because these techniques are arbitrary cycles, it's challenging to regulate the consistency and dispersion of nanostructures on the embedded surfaces. Scientists have devised a new covering strategy fueled by the regular biomineralization cycle. Precipitation of calcium phosphate apatite precious stones onto the Ti surface from reenacted body liquids (simulated body fluid (SBF)) framed a covering at room temperature in this biomimetic strategy. A few techniques have been developed to speed up the statement of coatings from watery arrangements (Shadanbaz et al., 2012; Bose et al., 2012). In preclinical relative models, the osseointegration of Ti inserts coated with biomimetic calcium phosphate has been studied (Habibovic et al., 2002, 2005). In any case, the osseointegration of biomimetic Ti dental inserts has yet to be compared to other surface medicines in preclinical models. Bone-invigorating agents, such as growth factors, could be applied outside of Ti dental inserts to improve the bone-recovery measure locally. Recent research has revealed that bioactive specialists may improve the embedded surface's osteogenic properties (Schwartz-Filho et al., 2012; Bougas et al., 2014). Bioactive inserts have been considered to create a biochemical bond between the bone tissue and the Ti-embedded surface rather than just a physical one (Sul et al., 2010). A bioactive embed surface can promote various sub-atomic collaborations, potentially forming a substantial connection between the bone and the embed surface (Sul et al., 2013). Fibronectin, fibroblast growth factor (FGF), type I collagen, Bone morphogenetic proteins (BMPs), and arginine-glycine-aspartic acid (RDG peptide) are promising bioactive sub-atomic up-and-comers with high osteogenic potential, according to a few studies (Jimbo et al., 2007).

A blend of RGD peptides (aspartate glycine and arginine) was used to create a lattice using acrylate stays and the Nano mechanical dock of collagen I filaments (Schliephake et al., 2008), causing increased bone-embed contact and bone thickness during the early stages of peri-embed bone development effectively after one month. With the ability to promote cell bonding via integrin transmembrane receptors important for cell-extracellular grid collaborations, arginyl glycyl aspartic corrosive tripeptide has been thoroughly researched in vitro and preclinical creature models (Hanawa et al., 2010). However, the cost of producing these bioactive particles and specialized and administrative issues have prompted researchers to investigate alternative bioactive atoms, like the bone-preparing hormone nutrient D (Kelly et al., 2009).

Amorphous material, diamond-like carbon (DLC), is used to coat dental implants by deposition of an intermediate layer for experimental study with high inherent biocompatibility with bone. This process is known as chemical vapor deposition (CVD) onto heated CPTi abutment screws and includes electrodeposition. DLC produces enhanced biocompatibility and improved corrosion resistance, with *in vitro* experimental indication of achievement. However, it requires *in vivo* despite this promise before clinical practice (patients) (Huacho et al., 2017). Hovsepian et al. (2022) reported the structural response and load-bearing capacity of TiN/NbN superlattice coatings deposited on medical-grade CoCrMo alloy substrate. The coatings were applied by a mixed High Power Impulse Magnetron Sputtering-Unbalanced Magnetron Sputtering (HIPIMS-UBM) process. The coated CoCrMo alloy was studied under localized load to investigate the crack formation mechanism. The high toughness of the superlattice structured TiN/NbN coatings was obtained, which, combined with their high adhesion on the substrate, made the coated medical grade CoCrMo alloy a potential candidate for medical implant applications.

Implant placement in dentistry and orthopedics focuses on improving the osseointegration and biocompatibility properties of Ti and Ti-based composites by the versatile surface modification layer-by-layer technique. In future applications in Ti-based composite implants, the morphology and chemical structure could be characterized by (i) ultraviolet-visible, (ii) atomic force microscopy, (iii) Fourier-transform infrared spectroscopies, (iv) scanning electron microscopy, and (v) micro-Raman spectroscopy. Films of poly (sodium 4-styrene sulfonate) (PSS) and Ti dioxide (TiO_2_) nanoparticles multilayers might enhance the screw topography and chemical surface properties with beneficial effects for osteoblast activity to improve dental implants (Igor et al., 2021).

## 11 Conclusions

In dentistry, Ti and Ti alloys are considered to be the materials of excellence due to their optimum physical, mechanical and biochemical properties. Because of the generally increased costs, handling of Ti and Ti alloys using advanced additive manufacturing (AM) was given insufficient attention by physicians until a few years ago. However, advanced AM methods like LMD, EBM, SLM etc. are getting progressively well-known in dental applications due to their ability to produce implants with customized designs and surface morphologies that allow easy cell multiplication required for bone ingrowth. Various advances have aided the osseointegration in physical and chemical surface modification approaches. However, still there is a great need for long-term clinical research to compare the performance of different coatings, and evaluate the success rate of innovative implant coatings. In conclusion, Ti and Ti alloys are anticipated to remain the mainstream implant materials in dentistry with the advancement of continual research.

## Declarations

### Author contribution statement

All authors listed have significantly contributed to the development and the writing of this article.

### Funding statement

This research did not receive any specific grant from funding agencies in the public, commercial, or not-for-profit sectors.

### Data availability statement

No data was used for the research described in the article.

### Declaration of interests statement

The authors declare no conflict of interest.

### Additional information

No additional information is available for this paper.
